# A Two-Stage Method of Dimensioning and Scheduling Service Providers under Patient Demand Uncertainty

**DOI:** 10.1155/2022/4377142

**Published:** 2022-10-05

**Authors:** Hajar Shirneshan, Ahmad Sadegheih, Hasan Hoseini Nasab, Mohammad Mehdi Lotfi

**Affiliations:** Yazd University, Yazd, Iran

## Abstract

Many researchers have studied the problem of dimensioning service providers and making shift schedules and have proposed various methods to solve it. Considering the importance and complexity of health care, this research is conducted through the integrated dimensioning and scheduling of service providers under patient demand uncertainty. In the first stage, a robust approach is adopted to determine the minimum number of required service providers. In the second stage, a monthly schedule is devised for service providers, and a two-stage stochastic program is used to solve the problem. To this end, an improved sample average approximation method considers different contracts and skills to determine a near-optimal schedule by minimizing the service providers' regular working hours, overtime, and penalties for idle hours. In the first stage, considering the highest level of conservatism, equal to 7.6, a 19.38% cost increase is created compared to the nominal problem. In the second stage, by applying different clustering methods in the SAA algorithm and comparing them, the k-means++ algorithm obtains a good upper and lower bound and achieves a near-optimal solution in the shortest time. This research deals with the Iranian Health Control Center as a case study. The proposed method can yield the appropriate number of service providers based on monthly workloads and make the least undesirable schedules for service providers. Hence, managers can overcome patient issues' uncertainty by assigning various service providers to each scheduling period.

## 1. Introduction

Due to the increase in chronic diseases such as cancer, diabetes, and COVID-19, the costs of healthcare systems are rising dramatically [1]. Alternatively, the population is aging, and more health services are needed with the baby boom generation entering middle age. In 2029, the last group of baby boomers will retire, resulting in a 73% increase in Americans aged 65 and older. Also, by 2050, one out of six people in the world will be over 65, while in 2019, it was one person out of eleven [2]. The statistics issued by the World Health Organization indicate that personnel planning will be a priority in the field of health in the next decade. Due to the high cost of staffing, which accounts for about 40% of the total costs, medical centers have to reduce their expenditures. Healthcare organizations face the question of how to organize the size and structure of their workforce to manage upcoming workloads more cost-effectively. This issue is especially the case when current and future demands deviate from each other. Cancer patients are among those who have this uncertain demand.

The dimensioning of service providers is no longer an easy task to service with only one type of service provider. It gets even more challenging with the heterogeneity of the workforce due to different types of skills or contracts [3]. Considering service providers' size and structure (e.g., skill sets and contract types), dimensioning aims to determine the adequate number needed in different categories. As another crucial task in service provider planning, scheduling involves getting the right service provider to the right shift on the right day. The nurse rostering problem (NRP), or nurse scheduling problem (NSP), aims to schedule and assign available service providers to hospital shifts under various constraints over a period [4]. It is easy to recognize that dimensioning decisions impact the scheduling quality directly. Hence, it is reasonable not to look at dimensioning and scheduling decisions as two consecutive tasks but to employ an integrated planning approach. As a result, dimensioning and scheduling service providers is a critical issue for health care centers. In the literature, there are few contributions addressing integrated dimensioning and scheduling compared to the literature on dimensioning or scheduling problems. Since health care centers have access to a limited number of service providers with certain contract and skill types, the proper dimensioning and planning of personnel gains importance. According to previous research, most researchers in this field have concentrated on staff dimensioning or scheduling issues with a specific number of service providers. However, due to the uncertainty of patient issues (such as the varied number of patients, different levels of patients' severity, and unpredictable patients' situations) or service provider issues (e.g., absence, pregnancy, and fatigue), health care centers require different numbers of service providers for certain planning periods (Tuna et al. [5]; Wang et al. [6]). Healthcare center managers should forecast and determine the future service providers' size based on uncertainty (Tuna et al. [5]) to ensure that they are flexible in assigning extra service providers to other departments or teams or requesting extra service providers from them, as necessary. Thus, a health care center manager should negotiate the size of the service providers before making a schedule. For example, in the Iranian health control center, due to the uncertainty in the conditions of cancer patients, determining the appropriate number of service providers is critical. Cancer patients experience sudden changes such as metastasis and lymphedema, which lead to uncertainty in their conditions. In the Iranian health control center, the contracts signed by service providers with different skills are set in three modes, namely, full-time, part-time, and hourly. The service cost increases by 20% to 40% per hour as a contract is changed from full-time to part-time or hourly. Therefore, planning for the proper assignment of service providers can significantly save system costs. As is the case, most health care centers use manual planning, and the Iranian health control center is no exception [7]. The present study focuses on providing specialized services to cancer patients in the event of demand uncertainty to address the issue of planning the service providers in this center.

Motivated by the previous research, this study proposes a method to evaluate the required service providers with different skills and contracts and make the corresponding schedule in an uncertain environment. So, the managers have the flexibility to reassign their service providers to other healthcare centers or get help from them to prepare care. This research integrates dimensioning and scheduling problems with patient demand uncertainty. Academic methods are lacking for dealing with such practical car providers' dimensioning and scheduling problems. This lack of methodology serves as the motivation for this research. To the best of our knowledge, B. Vanhoucke and M. Vanhoucke [8], Wright and Mahar [9], Chen et al. [10], and Respicio et al. [11] are the only researchers that have combined the dimensioning and scheduling issues of service providers to form an integrated service provider dimensioning and scheduling problem (ISPDSP). This new ISPDSP involves two decisions: (1) determining the size of the service providers at the beginning of each period and (2) creating a schedule based on that information. The present study aims to create a two-phase method that integrates a robust approach and two-stage stochastic programming to solve the ISPDSP. The presented method will help managers to determine the required number of service providers based on the conservatism level, which is determined according to the working conditions of the health center. Suppose the patients' conditions at the health center are such that the smallest delay in the service leads to the deterioration of the patient's condition. In that case, the level of conservatism is considered at its highest value. Next, based on a two-stage stochastic programming model, the shift planning of each service provider is determined.

## 2. Literature Review

Medical staff planning has been a topic of research since the 1950s. Ernst et al. [12] indicated that it is difficult to create a schedule that meets the needs of employees. The task of medical staff planning is often difficult due to staffing requirements as well as government and hospital regulations. Different subjects, such as the number and conditions of the patients, the medical staff's skills, preferences, and experiences, and government regulations should be considered by planners [12]. More studies on this issue have been published over the last two decades because of the significance of medical staff scheduling in healthcare.

Many articles have been reviewed about medical staff scheduling. Cheang et al. [13], Ernst et al. [12], Viana [14], Van den Bergh et al. [15], and Defraeye and Van Nieuwenhuyse [16] categorized medical staff scheduling problems based on their characteristics, solution methods, and future research trends. Klinz et al. [17] used two mathematical models to minimize the number of work shifts and nurses' general unhappiness. Topaloglu and Selim [18] proposed a multiobjective fuzzy goal programming model for NSPs. The model satisfies the hospital management objectives and makes an equitable schedule for nurses. They provided different fuzzy solution approaches to solve the problem. They studied the fulfilling demand coverage for the hospital's objective and satisfaction for nurses' objectives, which contains desired shift types, requested days off, work patterns, and total workload. Different types of membership functions, such as trapezoidal and triangular, were considered. Also, a sensitivity analysis is performed to provide decision-makers with a more confident solution set. Landa-Silva and Le [19] faced real-world uncertainties through a multiobjective approach to achieve high-quality nondominated schedules. They solved the model with a simple evolutionary algorithm. Ohki [20] established a cooperative genetic algorithm to reoptimize nurse schedules. Zhang et al. [21] presented a hybrid swarm-based optimization algorithm that combined a variable neighborhood search and a genetic algorithm to face highly constrained nurse scheduling problems in hospital environments. Maenhout and Vanhoucke [8] studied the nurse allocation issue and used the column-generation method to deal with it. Santos et al. [22] introduced cutting in integer programming to solve the problem involved innovatively. Ingels and Maenhout [23] introduced reserve duties and surveyed their impact on medium-term personnel shift rosters. They evaluate the delivered robustness by imitating the workforce management process in a three-step method. The unexpected events were simulated after designing the personnel roster. Finally, an optimization model determined the required adjustments to balance the supply and demand. Dohn and Mason [24] defined a generalized staff scheduling problem as containing a master problem and a subproblem. The master problem specified the roster lines of the staff to satisfy the demand constraints, and the subproblem generated a feasible roster line. Those researchers applied the branch-and-price concept and column-generation to solve the master problem and subproblems. Bagheri et al. [25] introduced a stochastic mathematical model for an NSP in the heart surgery department at Razavi Hospital to minimize the regular and overtime assignment costs. They assumed that patients' demands and length of stay would be uncertain. So, they used the sample average approximation method to solve the problem. Punnakitikashem et al. [26] used a stochastic integer MP model to minimize the overload of nurses. Staffing cost is considered through a hard budget constraint in the model. They used the Benders' decomposition and Lagrangian relaxation methods to achieve nondominated solutions. Northeast Texas Hospital is considered for implementing the introduced model as a case study. Chen et al. [10] studied an integrated problem of medical staff allocation and staff scheduling in uncertain environments. They used a two-stage algorithm based on goal programming and determined the smallest possible medical staff required to make the best schedule for them. Ang et al. [27] introduced a goal programming model for NSPs and developed a decision support system. They examined the workload distribution, shift equity, and staff satisfaction. They also pursued minimizing the nurse-patient ratio (NPR) and calculated it based on the number of patients allocated to each nurse. Hamid et al. [28] proposed a multiobjective mathematical model for nurse scheduling, which took the decision-making styles of nurses into account. The objectives addressed in that study were minimization of the average index of the incompatibility in the decision-making styles of the nurses assigned to the same shift days, maximization of the overall satisfaction of nurses with their shifts, and minimization of the total cost of staffing. Moreover, three meta-heuristics were developed to solve the problem, including multiobjective tabu search, the nondominated sorting genetic algorithm, and the multiobjective Keshtel algorithm. Pham and Dao [29] proposed a method by grouping nurses into clusters. Then, a hybrid metaheuristic algorithm consisting of the grey wolf optimizer (GWO) and particle swarm optimization (PSO) prepared the scheduling of each cluster. The results from the hybrid algorithm were compared to those from the standard PSO, GWO, and a linear programming formulation to evaluate the algorithm's effectiveness. Hassani and Behnamian [30] developed a sustainable approach with a robust scenario-based optimization method. They proposed the differential evolution (DE) algorithm to solve the problem and compared its performance to the genetic algorithm. The results show that the DE algorithm has good performance. Kheiri et al. [31] studied the multistage nurse rostering formulation. They proposed a sequence-based selection hyper-heuristic using a statistical Markov model and an algorithm for building feasible initial solutions. Empirical results and analysis show that the suggested approach has significant potential for difficult problem instances.

Many researchers have considered uncertainty regarding the patient, medical staff, or operational issues. Still, few have studied uncertainty regarding staff size when examining medical staff scheduling problems. Wang et al. [6] focused on a two-phase study of nurse scheduling. They employed forecasting technology during the first phase to predict the number of nurses required for the next four weeks. They used a two-cohort staggering strategy to schedule the required nurses for each shift on each day during the second phase. Tuna et al. [5] determined the required number of nurses in an outpatient chemotherapy unit for five consecutive weeks. They used historical data about the six kinds of patients and the average treatment time for each kind on a daily horizon. The results demonstrated that, based on the uncertainty in the patients' number and treatment time, the required number of nurses varied from day to day for the next five-week planning period, ranging from 6 to 32. Uno [32] dealt with a staff scheduling problem by calculating the size of the medical staff needed for home care. They determined the total required services for each period and used a mathematical model to calculate the lower and upper bounds of the helpers for each period.  Table 1 presents a brief classification of the models reviewed in the literature.

Based on these studies, the number of service providers changes from one period to another. Hence, this research employed a conservative service provider size to make a monthly schedule by considering the patient demand uncertainty. In real-world shift scheduling, a different source of uncertainties needs to be addressed to provide a reliable schedule. Therefore, this study presents a two-stage stochastic programming model that considers the uncertainty in patients' demands, types of contracts, and service providers' skills. In the following, the improved sample average approximation (I-SAA) method is employed to solve the model, and the parameters of the solution method are adjusted (Figure 1).

The rest of this article is as follows. The proposed optimization model and its structure are presented in Section 3.  Section 4 introduced the solution approach with detailed descriptions of the original SAA and I-SAA methods.  Section 5 presents numerical experiments. Finally, the concluding remarks are made in Section 6.

## 3. Problem Definition and Modeling

### 3.1. Service Providers Dimensioning Problem (SPDP)

The robust approach is suitable for dealing with uncertainty, which was first proposed by Soyster in the early 1970s [34]. In an uncertain environment, a range of possible values for key parameters can be related to the objective function or constraints. This range of values is specified as the lower and upper bounds for the main parameters, and robust optimization evaluates them. Then, a conservative level is selected as the predetermined value of each parameter, and the corresponding problem is formulated. Soyster [34] proposed a very conservative approach; therefore, the answer obtained is so far from the answer of the nominal model. Ben-Tal and Nemirovski [35] considered an ellipsoidal uncertainty set and presented a conic quadratic program that cannot be directly used for discrete models. Sim [36] presented a different approach for controlling the level of conservatism, which leads to a linear programming model. This formulation, called “budget of uncertainty,” allows a model's uncertainty to be adjusted based on the decision maker's risk adversity through an uncertainty budget and causes a small increase in computational efforts compared to deterministic approaches. So, the present study employed Bertsimas' approach to formulate deterministic MILPs into robust optimization counterparts. Therefore, mathematical programming can obtain optimal solutions to the corresponding problem. The most conservative response obtained from solving this model determines the number of service providers required, as presented in Section 3.2.  Table 2 presents the notations of SPDP.

Based on the problem uncertainties, the patients' demands and the contract duration for each skill vary from period to period. The parameters *d*_*im*_ and *ca*_*jm*_, independent of each other, have an unknown distribution but are symmetric in a range, possibly with an average equal to their nominal values. So, *d*_*im*_ and *ca*_*jm*_ take $\left[{d_{im}-{\hat{d}}_{im},d}_{im}+{\hat{d}}_{im}\right]$ and $\left[{{ca}_{jm}-{\hat{ca}}_{jm},ca}_{jm}+{\hat{ca}}_{jm}\right]$, where ${\hat{d}}_{im}$ and ${\hat{ca}}_{jm}$ represent the deviation from the nominal coefficients *d*_*im*_ and *ca*_*jm*_, respectively. To formulate the robust counterpart of the problem, Γ_*im*_, *i* ∈ *S*, *m* ∈ *M* values are defined for uncertain constraints. Thus, the goal is to find the optimal solution in situations with Γ_*im*_, *iϵ*{1,2,…, *S*}, *m* ∈ {1,2,…, *M*}. The details of how this formulation can be derived are presented in reference [37]. It is also shown that the resulting robust problem is solvable within a polynomial time. The robust model can be defined as follows:

(1) $$\begin{array}{c} \begin{array}{c} min\;\overset{S}{\underset{i=1}{\sum }}\overset{N}{\underset{j=1}{\sum }}\overset{M}{\underset{m=1}{\sum }}c_{ijm}x_{ijm}\\ \overset{N}{\underset{j=1}{\sum }}{ca}_{jm}x_{ijm}-\left[z_{im}\Gamma_{im}+{\sum p_{ijm}}_{j\in J_{i}}+p_{im0}\right]\geq d_{im}\forall i,\forall m \end{array}\text{,} \end{array}$$

(2) $$\begin{array}{c} z_{im}+p_{ijm}\geq {\hat{ca}}_{jm}\left|x_{ijm}\right|\forall j\in J_{i},\forall i,\forall m\text{,} \end{array}$$

(3) $$\begin{array}{c} z_{im}+p_{im0}\geq {\hat{d}}_{im}\forall i,\forall m\text{,} \end{array}$$

(4) $$\begin{array}{c} \overset{n}{\underset{j=1}{\sum }}x_{ijm}\leq a_{im}\;\forall i,\forall m\text{,} \end{array}$$

(5) $$\begin{array}{c} \overset{m}{\underset{i=1}{\sum }}x_{ijm}\leq b_{jm}\;\forall j,\forall m\text{,} \end{array}$$

(6) $$\begin{array}{c} \overset{n}{\underset{j=1}{\sum }}x_{ijm}\geq 1\;\forall i,\forall m\text{,} \end{array}$$

(7) $$\begin{array}{c} z_{im},p_{im0}\geq 0\forall i,\forall m\text{,} \end{array}$$

(8) $$\begin{array}{c} p_{ijm}\geq 0\forall i,\forall j,\forall m\text{ ,} \end{array}$$

(9) $$\begin{array}{c} x_{ijm}\epsilon \left\{0,1\right\}\forall i,\forall j,\forall m\text{.} \end{array}$$

The objective function minimizes the cost of the required service providers. Constraints (1), (2), and (3) guarantee the meeting of the demands for each month and each skill under robust optimization. Constraint (4) limits the number of service providers per skill. Constraint (5) limits the number of service providers per contract. Constraint (6) indicates that at least one service provider of each skill must be assigned each month. After the number of the required service providers is determined, nurse scheduling is addressed in Section 3.2.

### 3.2. Stochastic Service Providers' Scheduling Problem (SSPSP)

The proposed mathematical model assigns service providers to shifts, and the number of required overtime and idle hours in possible conditions is determined. The required duration of each skill per shift and per day (*de*_*sm* *d*_) is considered stochastic. Service providers are categorized into nurses, general practitioners, and specialists depending on their skills. Contracts are also available in full-time, part-time, and hourly types, 8, 4, and 2 hours per shift, respectively.  Table 3 presents the notations used in the model.

The stochastic demand model for the service providers' scheduling problem can be formulated as follows:

(10) $$\begin{array}{c} \mathrm{Min}\;Z=\overset{D}{\underset{d=1}{\sum }}\overset{M}{\underset{m=1}{\sum }}\overset{I_{xx}}{\underset{i=1}{\sum }}\overset{N}{\underset{j=1}{\sum }}{h_{j}ca}_{j}{aa}_{ij}{xx}_{imd}+\overset{D}{\underset{d=1}{\sum }}\overset{M}{\underset{m=1}{\sum }}\overset{I_{xy}}{\underset{i=1}{\sum }}\overset{N}{\underset{j=1}{\sum }}{h_{j}cb}_{j}{ab}_{ij}{xy}_{imd}+\overset{D}{\underset{d=1}{\sum }}\overset{M}{\underset{m=1}{\sum }}\overset{I_{xz}}{\underset{i=1}{\sum }}\overset{N}{\underset{j=1}{\sum }}{h_{j}cc}_{j}{ac}_{ij}{xz}_{imd}+\underset{\xi \epsilon B}{\sum }\overset{D}{\underset{d=1}{\sum }}\overset{M}{\underset{m=1}{\sum }}\underset{i\epsilon S}{\sum }\phi \left(\xi \right)\left(c1ip_{imd}^{\xi }+{c2}_{i}q_{imd}^{\xi }\right), \end{array}$$

(11) $$\begin{array}{c} \overset{M}{\underset{m=1}{\sum }}{xx}_{imd}\leq 1\text{,}\\ d=1,..,D\text{,} \end{array}$$

(12) $$\begin{array}{c} \overset{M}{\underset{m=1}{\sum }}{xy}_{imd}\leq 1\text{,}\\ i=1,\ldots ,I_{xy}\text{,}\\ d=1,..,D\text{,} \end{array}$$

(13) $$\begin{array}{c} \overset{M}{\underset{m=1}{\sum }}{xz}_{imd}\leq 1\text{,}\\ i=1,\ldots ,I_{xz}\text{,}\\ d=1,..,D\text{,} \end{array}$$

(14) $$\begin{array}{c} {xx}_{i3\;d}+{xx}_{ij\left(d+1\right)}\leq 1i=1,\ldots ,I_{xx,\;}d=1,..,D-1\;j=1,\ldots ,M\text{,} \end{array}$$

(15) $$\begin{array}{c} {xy}_{i3\;d}+{xy}_{ij\left(d+1\right)}\leq 1\;i=1,\ldots ,I_{xy},d=1,..,D-1\;j=1,\ldots ,M\text{,} \end{array}$$

(16) $$\begin{array}{c} {xz}_{i3\;d}+{xz}_{ij\left(d+1\right)}\leq 1\;i=1,\ldots ,I_{xz},d=1,..,D-1\;j=1,\ldots ,M\text{,} \end{array}$$

(17) $$\begin{array}{c} \overset{D}{\underset{d=1}{\sum }}\overset{M}{\underset{m=1}{\sum }}\left({1-xx}_{imd}\right)g_{d}\geq n1\;i=1,\ldots ,I_{xx}\text{,} \end{array}$$

(18) $$\begin{array}{c} \overset{D}{\underset{d=1}{\sum }}\overset{M}{\underset{m=1}{\sum }}\left({1-xy}_{imd}\right)g_{d}\geq n1\;i=1,\ldots ,I_{xy}\text{,} \end{array}$$

(19) $$\begin{array}{c} \overset{D}{\underset{d=1}{\sum }}\overset{M}{\underset{m=1}{\sum }}\left({1-xz}_{imd}\right)g_{d}\geq n1\;i=1,\ldots ,I_{xz}\text{,} \end{array}$$

(20) $$\begin{array}{c} \overset{D}{\underset{d=1}{\sum }}{xx}_{i3\;d}\leq n2,\;i=1,\ldots ,I_{xx}\text{ ,} \end{array}$$

(21) $$\begin{array}{c} \overset{D}{\underset{d=1}{\sum }}{xy}_{i3\;d}\leq n2,\;i=1,\ldots ,I_{xy}\text{,} \end{array}$$

(22) $$\begin{array}{c} \overset{D}{\underset{d=1}{\sum }}{xz}_{i3\;d}\leq n2,\;i=1,\ldots ,I_{xz}\text{,} \end{array}$$

(23) $$\begin{array}{c} {wx}_{id}=\overset{M}{\underset{m=1}{\sum }}{xx}_{imd},\;i=1,\ldots ,I_{xx},\;d=1,..,D\text{,} \end{array}$$

(24) $$\begin{array}{c} {wy}_{id}=\overset{M}{\underset{m=1}{\sum }}{xy}_{imd},\;i=1,\ldots ,I_{xy},\;d=1,..,D\text{,} \end{array}$$

(25) $$\begin{array}{c} {wz}_{id}=\overset{M}{\underset{m=1}{\sum }}{xz}_{imd},\;i=1,\ldots ,I_{xz},\;d=1,..,D\text{,} \end{array}$$

(26) $$\begin{array}{c} {wx}_{id}+\overset{n3}{\underset{t=1}{\sum }}{wx}_{i\left(d+t\right)}\leq n3\;i=1,\ldots ,I_{xx},d=1,..,D-n3+1\text{ ,} \end{array}$$

(27) $$\begin{array}{c} {wy}_{id}+\overset{n3}{\underset{t=1}{\sum }}{wy}_{i\left(d+t\right)}\leq n3\;i=1,\ldots ,I_{xy},d=1,..,D-n3+1\text{ ,} \end{array}$$

(28) $$\begin{array}{c} {wz}_{id}+\overset{n3}{\underset{t=1}{\sum }}{wz}_{i\left(d+t\right)}\leq n3\;i=1,\ldots ,I_{xz},d=1,..,D-n3+1\text{ ,} \end{array}$$

(29) $$\begin{array}{c} \overset{D}{\underset{d=1}{\sum }}\overset{M}{\underset{m=1}{\sum }}{{aa}_{ij}xx}_{imd}\geq {e1}_{xx}\;j=1,i=1,\ldots ,I_{xx}\text{,} \end{array}$$

(30) $$\begin{array}{c} \overset{D}{\underset{d=1}{\sum }}\overset{M}{\underset{m=1}{\sum }}{{ab}_{ij}xy}_{imd}\geq {e1}_{xy}\;j=1,i=1,\ldots ,I_{xy}\text{,} \end{array}$$

(31) $$\begin{array}{c} \overset{D}{\underset{d=1}{\sum }}\overset{M}{\underset{m=1}{\sum }}{{ab}_{ij}xz}_{imd}\geq {e1}_{xz}\;j=1,i=1,\ldots ,I_{xz}\text{,} \end{array}$$

(32) $$\begin{array}{c} \overset{D}{\underset{d=1}{\sum }}\overset{M}{\underset{m=1}{\sum }}{{aa}_{ij}xx}_{imd}\leq {e2}_{xx}\;j=1,i=1,\ldots ,I_{xx}\text{,} \end{array}$$

(33) $$\begin{array}{c} \overset{D}{\underset{d=1}{\sum }}\overset{M}{\underset{m=1}{\sum }}{{ab}_{ij}xy}_{imd}\leq {e2}_{xy}\;j=1,i=1,\ldots ,I_{xy}\text{,} \end{array}$$

(34) $$\begin{array}{c} \overset{D}{\underset{d=1}{\sum }}\overset{M}{\underset{m=1}{\sum }}{{ab}_{ij}xz}_{imd}\leq {e2}_{xz}\;j=1,i=1,\ldots ,I_{xz}\text{,} \end{array}$$

(35) $$\begin{array}{c} p_{\left(xx\right)m\;d}^{\xi }\geq {de}_{\left(xx\right)m\;d}^{\xi }-\overset{N}{\underset{j=1}{\sum }}\overset{I_{xx}}{\underset{i=1}{\sum }}{{h_{j}aa}_{ij}xx}_{imd}\;m=1,2,3,d=1,\ldots ,D\text{,} \end{array}$$

(36) $$\begin{array}{c} p_{\left(xy\right)m\;d}^{\xi }\geq {de}_{\left(xy\right)m\;d}^{\xi }-\overset{N}{\underset{j=1}{\sum }}\overset{I_{xy}}{\underset{i=1}{\sum }}{{h_{j}ab}_{ij}xy}_{imd}\;m=1,2,3,d=1,\ldots ,D\text{,} \end{array}$$

(37) $$\begin{array}{c} p_{\left(xz\right)m\;d}^{\xi }\geq {de}_{\left(xz\right)m\;d}^{\xi }-\overset{N}{\underset{j=1}{\sum }}\overset{I_{xz}}{\underset{i=1}{\sum }}{{h_{j}ab}_{ij}xz}_{imd}\;m=1,2,3,d=1,\ldots ,D\text{,} \end{array}$$

(38) $$\begin{array}{c} q_{\left(xx\right)m\;d}^{\xi }\geq {\overset{N}{\underset{j=1}{\sum }}\overset{I_{xx}}{\underset{i=1}{\sum }}{{h_{j}aa}_{ij}xx}_{imd}-de}_{\left(xx\right)m\;d}^{\xi }\;m=1,2,3,d=1,\ldots ,D\text{,} \end{array}$$

(39) $$\begin{array}{c} q_{\left(xy\right)m\;d}^{\xi }\geq {\overset{N}{\underset{j=1}{\sum }}\overset{I_{xy}}{\underset{i=1}{\sum }}{{h_{j}aa}_{ij}xy}_{imd}-de}_{\left(xy\right)m\;d}^{\xi }\;m=1,2,3,d=1,\ldots ,D\text{,} \end{array}$$

(40) $$\begin{array}{c} q_{\left(xz\right)m\;d}^{\xi }\geq {\overset{N}{\underset{j=1}{\sum }}\overset{I_{xz}}{\underset{i=1}{\sum }}{{h_{j}aa}_{ij}xz}_{imd}-de}_{\left(xz\right)m\;d}^{\xi }\;m=1,2,d=1,\ldots ,D\text{,} \end{array}$$

(41) $$\begin{array}{c} {xx}_{imd}\;\epsilon \left\{0,1\right\}m=1,2,3,d=1,\ldots ,D,i=1,\ldots ,I_{xx}\text{,} \end{array}$$

(42) $$\begin{array}{c} {xy}_{imd}\;\epsilon \left\{0,1\right\}m=1,2,3,d=1,\ldots ,D,i=1,\ldots ,I_{xy}\text{,} \end{array}$$

(43) $$\begin{array}{c} {xz}_{imd}\;\epsilon \left\{0,1\right\}m=1,2,3,d=1,\ldots ,D,\;i=1,\ldots ,I_{xz}\text{,} \end{array}$$

(44) $$\begin{array}{c} p_{imd}^{\xi },q_{imd}^{\xi }\geq 0\;i\in S\;,\xi \in B\text{,} \end{array}$$

The objective function minimizes regular work hours, overtime hours, and the cost of idle hours. In this regard, *ϕ*(*ξ*) is the probability of scenario *ξ*=1,2,…, *B* and ∑_*ξϵB*_*ϕ*(*ξ*)=1. Constraints (11)–(13) ensure that each nurse, general practitioner, and specialist is assigned a maximum of one shift per day. Constraints (14)–(16) state that if a service provider is assigned to a night shift, he or she should not work the following day. Constraints (17)–(19) specify that each service provider be assigned at least n1 weekend. Constraints (20)–(22) determine the maximum number of night shifts per service provider. Constraints (23)–(26) indicate that a service provider cannot work for more than *n*3 consecutive days. Constraints (27)–(29) state that each service provider with a full-time contract must work at least one *e*1_*i*_ shifts during the planning period. Constraints (30)–(32) limit the maximum number of shifts per full-time service provider (*e*2_*i*_ ) in the planning period. Constraints (32)–(34) determine overtime hours for nurses, general practitioners, and specialists per shift in each scenario, respectively. Constraints (35)–(37) specify extra hours for nurses, general practitioners, and specialists per shift in each scenario, respectively. Eventually, constraints (38)–(40) define the model's variables. This research assumes that the required hours of practicing skills on shift *m* per day (*de*_*sm* *d*_) has a uniform distribution in the interval (a, b). An exact solution can be obtained for small-sized problems, but as the size of the problem increases, the solution time increases too. This study solves the SSPSP with an improved sample average approximation algorithm. A recourse action model is applied to formulate the model of solving the problem with that algorithm.  Section 3.3 delineates the basic properties of the new formulation [36].

### 3.3. Stochastic Integer Programming with a Recourse Model

Stochastic programming models have appeared as extensions of optimization problems with random parameters. Consider the optimization problem below[36]:

(45) $$\begin{array}{c} \min\;cx\text{,}\\ s.t.Ax=b\text{,}\\ Tx=h\text{,}\\ x\in X\text{,}\\ x\geq 0\text{.} \end{array}$$

In this model, *x* is the vector of decision variables, *Ax*=*b* are deterministic constraints, and **T***x*=**h** are uncertain constraints that the parameters **T** and **h** depend on information and become available only after a decision is made on *x*. A class of stochastic programming models, known as recourse models, is obtained by allowing additional or recourse decisions after realizing the random variables **T** and **h**. So, recourse models are dynamic; the stages model the time discretely based on the available data. If all the uncertainty is dissolved, a recourse model captures it with two stages, namely, “present” and “future.” Given a first-stage decision *x*, for every possible (**q**, **T**, **h**) realized as (*q*, *T*, *h*), the infeasibilities *h* − *Tx* are compensated at minimal costs with second-stage decisions as an optimal solution of the second-stage problem. This specifies the minimal recourse costs as a function of the first-stage decision *x*, and the realization of *ξ* is denoted by *υ*(*x*, *ξ*). Its expectation, *Q*(*x*)=*𝔼*_*ξ*_[*υ*(*x*, *ξ*)], yields the expected recourse costs associated with the first-stage decision *x*. Thus, the two-stage recourse model is as follows:

(46) $$\begin{array}{c} \min\;cx+Q\left(x\right)\text{,}\\ s.t.Ax=b\text{,}\\ x\in X\text{,} \end{array}$$

where the objective function *cx*+*Q*(*x*) indicates the total expected costs of decision *x* [36]. The SSPSP's first stage decisions include assigning service providers to work shifts. The decisions of the second stage are determined based on the stochastic demand of the patients. The following recourse model defines the stochastic model for the service providers' scheduling problem:

(47) $$\begin{array}{c} \begin{array}{cc} \mathrm{Min}\;Z=\overset{D}{\underset{d=1}{\sum }}\overset{M}{\underset{m=1}{\sum }}\overset{I_{xx}}{\underset{i=1}{\sum }}\overset{N}{\underset{j=1}{\sum }}{h_{j}ca}_{j}{aa}_{ij}{xx}_{imd}+\overset{D}{\underset{d=1}{\sum }}\overset{M}{\underset{m=1}{\sum }}\overset{I_{xy}}{\underset{i=1}{\sum }}\overset{N}{\underset{j=1}{\sum }}{h_{j}cb}_{j}{ab}_{ij}{xy}_{imd}+ & \overset{D}{\underset{d=1}{\sum }}\overset{M}{\underset{m=1}{\sum }}\overset{I_{xz}}{\underset{i=1}{\sum }}\overset{N}{\underset{j=1}{\sum }}{h_{j}cc}_{j}{ac}_{ij}{xz}_{imd}+E\left[Q\left(x,\xi \right)\right]. \end{array} \end{array}$$

Constraints (11)–(34):

In this model, *E*[*Q*(*x*, *ξ*)] shows the recourse action function, and

(48) $$\begin{array}{c} Q\left(x,\xi \right)=\min\underset{\xi \epsilon B}{\sum }\overset{D}{\underset{d=1}{\sum }}\overset{M}{\underset{m=1}{\sum }}\underset{i\epsilon S}{\sum }\phi \left(\xi \right)\left({c1}_{i}p_{imd}^{\xi }+{c2}_{i}q_{imd}^{\xi }\right). \end{array}$$

Constraints (35)–(40):

The *ξ* ∈ *B* vector contains numerous scenarios. So, to obtain *E*[*Q*(*x*, *ξ*)], lots of similar integer linear programs (ILPs) [38] must be solved, which is a difficult calculation task. Since it is hard to provide an exact solution to the SSPSP, the next section proposes an approximation.

## 4. Solution Approach

This research expands on a two-stage method to solve an ISPDSP. The Bertsimas approach (see Section 3.1) describes an SPDP based on the patients' demand uncertainty in the first step. Step two is calculating the minimum number of service providers required under budget uncertainty. In the third step, that minimum number serves as a basis to determine the final number of the service providers and to construct an SSPSP based on this number. The objective function of the SSPSP is to minimize the regular working hours, overtime hours, and penalty for idle hours costs. In the last step, the original SAA and I-SAA methods are employed to solve the SSPSP. This yields a near-optimal schedule for service providers. Solving the model can help managers determine appropriate service providers and make the corresponding schedules in uncertain environments.

### 4.1. The Sample Average Approximation (SAA)

There are several solution methods, such as the SAA to solve stochastic models. The SAA method solves stochastic programming problems based on the Monte Carlo simulation method. It generates a random sample and approximates the expected value function with the corresponding sample average function. The stop criterion determines how long the algorithm will last. Over the years, various authors have employed the idea of sample average approximation to solve stochastic programs. For example, it was employed to solve stochastic knapsack problems [39], stochastic routing problems [40], supply chain problems [41], and investment problems [42]. Due to the high applicability of the SAA method, it has been selected to solve the model in this study. The method is delineated below.

Let *M*, *N*, and *N*′ be the number of replications, the number of scenarios in the sample problem, and the sample size used to estimate $C^{T}\hat{x}+E\left[Q\left(\hat{X},\xi \right)\right]$ for a given feasible solution $\hat{x}$, respectively. So, the SAA method can be described as follows [40]:

(1) For *m* = 1,..., *M*, repeat the following steps:
  (a) Generate N random sample *ξ*^1^, *ξ*^2^ ,…, *ξ*^N^.
  (b) Solve the problem by the SAA method and let ${\hat{X}}_{N}^{m}$ be the solution vector and ${\hat{Z}}_{N}^{m}$ the optimal objective value.
  (c) Generate independent random sample *ξ*^1^, *ξ*^2^ ,…, *ξ*^*N*′^. Evaluate ${\hat{g}}_{N^{\prime }}\left({\hat{X}}_{N}^{m}\right)$ and $S_{{\hat{g}}_{N^{\prime }}\left({\hat{X}}_{N}^{m}\right)}^{2}$ as follows:
    (49) $$\begin{array}{c} {\hat{g}}_{N^{\prime }}\left({\hat{X}}_{N}^{m}\right)=\overset{D}{\underset{d=1}{\sum }}\overset{M}{\underset{m=1}{\sum }}\overset{I_{xx}}{\underset{i=1}{\sum }}\overset{N}{\underset{j=1}{\sum }}{h_{j}ca}_{j}{aa}_{ij}{xx}_{imd}+\overset{D}{\underset{d=1}{\sum }}\overset{M}{\underset{m=1}{\sum }}\overset{I_{xy}}{\underset{i=1}{\sum }}\overset{N}{\underset{j=1}{\sum }}{h_{j}cb}_{j}{ab}_{ij}{xy}_{imd}+\overset{D}{\underset{d=1}{\sum }}\overset{M}{\underset{m=1}{\sum }}\overset{I_{xz}}{\underset{i=1}{\sum }}\overset{N}{\underset{j=1}{\sum }}{h_{j}cc}_{j}{ac}_{ij}{xz}_{imd}+\frac{1}{N^{\prime }}\overset{N^{\prime }}{\underset{n=1}{\sum }}\overset{D}{\underset{d=1}{\sum }}\overset{M}{\underset{m=1}{\sum }}\underset{i\epsilon S}{\sum }\phi \left(\xi \right)\left({c1}_{i}p_{imd}^{\xi }+{c2}_{i}q_{imd}^{\xi }\right). \end{array}$$
    (50) $$\begin{array}{c} S_{{\hat{g}}_{N^{\prime }}\left({\hat{X}}_{N}^{m}\right)}^{2}=\frac{1}{N^{\prime }\left(N^{\prime }-1\right)}\overset{N^{\prime }}{\underset{n=1}{\sum }}\left[\left.\overset{D}{\underset{d=1}{\sum }}\overset{M}{\underset{m=1}{\sum }}\overset{I_{xx}}{\underset{i=1}{\sum }}\overset{N}{\underset{j=1}{\sum }}{h_{j}ca}_{j}{aa}_{ij}{xx}_{imd}+\overset{D}{\underset{d=1}{\sum }}\overset{M}{\underset{m=1}{\sum }}\overset{I_{xy}}{\underset{i=1}{\sum }}\overset{N}{\underset{j=1}{\sum }}{h_{j}cb}_{j}{ab}_{ij}{xy}_{imd}+\overset{D}{\underset{d=1}{\sum }}\overset{M}{\underset{m=1}{\sum }}\overset{I_{xz}}{\underset{i=1}{\sum }}\overset{N}{\underset{j=1}{\sum }}{h_{j}cc}_{j}{ac}_{ij}{xz}_{imd}+\overset{D}{\underset{d=1}{\sum }}\overset{M}{\underset{m=1}{\sum }}\underset{i\epsilon S}{\sum }{\phi \left(\xi \right)\left(c\right.1}_{i}p_{imd}^{\xi }+{c2}_{i}\left.q_{imd}^{\xi }\right)-{\hat{g}}_{N^{\prime }}\left(\bar{X}\right.\right)\right]\text{,} \end{array}$$
(2) Evaluate ${\bar{Z}}_{N}^{M}$ and $S_{{\bar{Z}}_{N}^{M}}^{2}$.
  (51) $$\begin{array}{c} {\bar{Z}}_{N}^{M}=\frac{1}{M}\overset{M}{\underset{m=1}{\sum }}{\hat{Z}}_{N}^{m}\;,S_{{\bar{Z}}_{N}^{M}}^{2}=\frac{1}{\left(M-1\right)M}{\overset{M}{\underset{m=1}{\sum }}\left[{\hat{Z}}_{N}^{m}-{\bar{Z}}_{N}^{M}\right]}^{2}\text{,} \end{array}$$
The confidence interval for the optimality gap can be calculated as follows:
  (52) $$\begin{array}{c} {\hat{g}}_{N^{\prime }}\left({\hat{X}}_{N}^{m}\right)-{\bar{Z}}_{N}^{M}+Z_{\alpha }{\left\{S_{{\hat{g}}_{N^{\prime }}\left(\bar{X}\right)}^{2}+S_{{\bar{Z}}_{N}^{M}}^{2}\right\}}^{0.5}\text{,} \end{array}$$
Here is *Z*_*α*_=Φ^−1^(1 − *α*), where Φ(**Z**) is the cumulative distribution of the standard normal distribution.
(3) For each solution ${\hat{X}}_{N}^{m}$, *m* = 1,...,M, estimate the optimality gap by ${\hat{g}}_{N^{\prime }}\left({\hat{X}}_{N}^{m}\right)-{\bar{Z}}_{N}^{M}$, along with an estimated variance of $S_{{\hat{g}}_{N^{\prime }}\left({\hat{X}}_{N}^{m}\right)}^{2}+S_{{\bar{Z}}_{N}^{M}}^{2}$. Choose one of the *M* candidate solutions based on the least estimated objective value.

In the algorithm, ${\bar{Z}}_{N}^{M}$ and ${\hat{g}}_{N^{\prime }}\left({\hat{X}}_{N}^{m}\right)$ are the lower bound (LB) and the upper bound (UB) of the optimal value, respectively [43]. The parameter ${\bar{Z}}_{N}^{M}$ shows an unbiased estimator of the optimal objective function $E\left({\hat{Z}}_{N}\right)$. Here,${\bar{Z}}_{N}^{M}=E\left({\hat{Z}}_{N}\right)$ and $E\left({\hat{Z}}_{N}\right)\leq Z^{*}$. Moreover, ${\hat{g}}_{N^{\prime }}\left({\hat{X}}_{N}^{m}\right)$ presents an unbiased estimator of the objective value $E\left({\hat{Z}}_{N}\right)$, but $E\left({\hat{g}}_{N^{\prime }}\left({\hat{X}}_{N}^{m}\right)\right)\geq Z^{*}$. An increase in the value of *N* causes an increase in the accuracy of the response as well as an exponential rise in the solution time [40]. Thus, by selecting sample size *N*, there is a trade-off between the computational complexity and the qualities obtained through solving the problem. The next section introduces clustering as one of the proposed methods to reduce the number of scenarios.

### 4.2. Clustering Techniques in Sample Average Approximation

In real-world situations with large problems, the SAA algorithm performs well, but the computation time is long and the method is inefficient. So far, just a few studies have been conducted on scenario clustering to solve optimization problems. Those who have tried to resolve this issue use clustering algorithms to group similar scenarios and generate samples. Crainic et al. [44] grouped progressive hedging algorithm scenarios by a machine learning method and applied the approach to a stochastic network design problem. They used clustering techniques inside a partial Benders decomposition algorithm to reduce the number of feasibility and optimality cuts generated by the algorithm. Emelogu et al. [45] employed clustering techniques to improve the SAA algorithm. They update the sample sizes dynamically and make high-quality solutions within a reasonable time. Sim [36] focused on clustering algorithms to categorize scenarios before selecting a random sample for the SAA algorithm. They extracted the data from a facility location problem. Clustering is the unsupervised classification that divides data into groups of similar objects [46]. Each group is called a cluster that contains similar data. Clustering algorithms are divided into three main categories: (1) partitional clustering; (2) hierarchical clustering; and (3) density-based clustering. Partitional clustering methods are divided into two subcategories, namely, centroid and medoid. The centroid algorithm specifies each cluster based on the gravity center of instances. Each cluster consists of the instances closest to the gravity center in the medoid algorithm. In this method, the numbers of the clusters are determined in advance. The hierarchical clustering method builds a tree of clusters known as a dendrogram that organizes clusters from the top-down. The density-based clustering algorithm determines the number of clusters automatically. This method divides data based on different criteria, such as connectivity, boundary, and region. Since in this research, clustering is done for different scenarios of patients' demand and the number of clusters is determined in advance, partitional clustering methods (e.g., K-means, K-means++, PAM, and EM-GMM) have been used for clustering the scenarios for the SAA algorithm. Then, a lower bound for the problem is obtained through the clustered scenarios.  Figure 2(a) shows all the possible scenarios generated by a stochastic program in a solution space. The original SAA takes a few scenarios as samples (*N*) from all the possible ones and calculates the objective function iteratively until *M* solutions are obtained. However, I-SAA groups the scenarios in the form of a cluster where each scenario highly represents that cluster (Figure 2(b)). The number of the scenarios (*N*_*k*_) for the I-SAA algorithm is the reduced form of each cluster (Figure 2(c)) [45].

The implementation of the I-SAA method is summed up as follows:

(1) For *m* = 1, ..., *M*, repeat the steps below:
  (a) Generate *N*_*L*_ random sample *ξ*^1^, *ξ*^2^,…, *ξ*^N_L_^(N_L_ ≫ N).
  (b) Use one of the clustering techniques described in Section and cluster N_L_ samples to yield N_k_ scenario.
  (c) Solve the problem by the I-SAA method and let ${\hat{X}}_{N_{k}}^{m}$ be the solution vector and ${\hat{Z}}_{N_{k}}^{m}$ the optimal objective value.
  (d) Generate an independent random sample *ξ*^1^, *ξ*^2^ ,…, *ξ*^*N*′^(*N*′ ≫ *N*_*L*_). Evaluate ${\hat{g}}_{N^{\prime }}\left({\hat{X}}_{N_{k}}^{m}\right)$ and $S_{{\hat{g}}_{N^{\prime }}\left({\hat{X}}_{N_{k}}^{m}\right)}^{2}$.
(2) Evaluate ${\bar{Z}}_{N_{k}}^{M}$ and $S_{{\bar{Z}}_{N_{k}}^{M}}^{2}$.
  (53) $$\begin{array}{c} {\bar{Z}}_{N_{k}}^{M}=\frac{1}{M}\overset{M}{\underset{m=1}{\sum }}{\hat{Z}}_{N_{k}}^{m}\;,S_{{\bar{Z}}_{N_{k}}^{M}}^{2}=\frac{1}{\left(M-1\right)M}{\overset{M}{\underset{m=1}{\sum }}\left[{\hat{Z}}_{N_{k}}^{m}-{\bar{Z}}_{N_{k}}^{M}\right]}^{2}\text{.} \end{array}$$
(3) Estimate the optimality gap ${\hat{g}}_{N^{\prime }}\left({\hat{X}}_{N_{k}}^{m}\right)-{\bar{Z}}_{N_{k}}^{M}$ for each solution ${\hat{X}}_{N_{k}}^{m}$ and the estimated variance of $S_{{\hat{g}}_{N^{\prime }}\left({\hat{X}}_{N_{k}}^{m}\right)}^{2}+S_{{\bar{Z}}_{N_{k}}^{M}}^{2}$, *m* = 1, ..., *M*. Choose one of the *M* candidate solutions based on the least estimated objective value.

Sections 4.2.1to 4.2.4 describe these clustering methods used in the original SAA algorithm.

#### 4.2.1. K-Means

Lloyd [47] proposed the K-means algorithm in 1957. Sometimes referred to as the Lloyd's algorithm, K-means is an easy, simple, efficient, and the most popular unsupervised learning algorithm used to classify a given dataset into a certain number of clusters in such a way that each dataset belongs to one cluster with the same properties. It has two phases. The first phase chooses the initial *k* centers at random. The second phase assigns each point in the dataset to the cluster consisting of the nearest center and determines each cluster's center value. Depending upon the new values of the centers, the second phase repeats until those values converge to the same value. Some of the important features of the K-means algorithm are being a common, fast, and well-known algorithm. It reaches convergence quickly because of its simplicity. Algorithm 1 demonstrates the steps of the K-means clustering algorithm.

#### 4.2.2. K-Means++

Although the K-means clustering algorithm is fast and simple in practice, recent works have mainly focused on improving the initialization procedure. Finding a better way to initialize the clusters, changes Lloyd's iteration's performance, and improve quality and convergence properties. Ostrovsky et al. [48] found that a simple procedure of selecting a good starting point could provide a good theoretical guarantee for the quality of the solution. They named this method the K-means++ clustering algorithm. The superiority of the K-means++ to the K-means clustering algorithm is implementing a better initialization approach to select the first k centers. In contrast to the K-means algorithm, the K-means++ algorithm only selects one cluster randomly. The remaining (k-1) centers are chosen systematically with a probability that is proportional to their contribution to the overall error. According to various datasets, the K-means++ algorithm makes considerable improvements compared to the K-means clustering algorithm, randomly selecting the centers. The steps involved in K-means++ clustering algorithm are illustrated in Algorithm 2.

#### 4.2.3. Expectation-Maximization Using Gaussian Mixture Models (EM-GMM)

The Gaussian mixture models (GMMs) consider the Gaussian distribution of clusters so that a cluster can be described by its mean and standard deviation [49]. GMMs are more flexible than K-means because they assume that clusters are Gaussian, while the K-means algorithm considers them circular. The parameters of the Gaussian distribution for each cluster are applied to optimize the EM (expectation-maximization) algorithm. The E-step in the EM algorithm focuses on probability estimation and parameter initialization. Then, the M-step maximizes the parameters through the probability estimates calculated in the E-step. The steps for the EM-GMM algorithm are outlined in Algorithm 3.

#### 4.2.4. Partitioning around Medoids (PAM)

The K-medoids algorithm is a modified version of the K-means algorithm. The K-medoids and K-means algorithms partition the dataset into groups and explore to minimize squared errors, which calculate the distance between the point designated as the center of that cluster and the points labeled to be in a cluster. The K-medoids algorithm chooses data points as centers, in contrast to the K-means algorithm. One of the best-known versions of K-medoids is PAM. It is a kind of iterative optimization that combines relocating the points between perspective clusters with renominating them as potential medoids [50]. A medoid can be specified as the object of a cluster whose average dissimilarity to all the objects in the cluster is minimal (i.e., it is the most centrally located point in a given dataset). The PAM algorithm operates in several steps. At first, the algorithm randomly selects *k* of the *n* data points as the medoids. Then, it associates each data point with the closest medoid by considering a distance method (e.g., Euclidean distance, Manhattan distance, and Minkowski distance). After that, the algorithm swaps each medoid and nonmedoid data point and computes the total cost of the configuration. Next, the lowest cost option is selected. Finally, the algorithm repeats until there is no change in the medoid. Algorithm 4 shows the steps of the PAM algorithm.

## 5. Numerical Experiments

### 5.1. Example Data

This section reports a case study planned at the Iranian Health Control Center, which provides palliative services to cancer patients. It currently serves about 370 patients. Before doing this research, planning was done manually by a care facilitator. Manual planning is very time-consuming, and it is not possible to take into account all the limitations. Therefore, the data are based on the Iranian Health Control Center, which can help with better planning in this center. Service providers with different skills, including nurses, general practitioners, and specialists, work in this center for 24 working days a month. Each day contains morning, afternoon, and night shifts. For the first model, the rate of the change in *d*_*im*_ and *ca*_*jm*_ is 5% of the nominal value. The corresponding data are obtained from the Iranian Health Control Center to evaluate the distribution of the demand for each skill per day and shift. The demand has a uniform distribution in the intervals of (24, 56), (12, 32), and (6, 14) per hour for nurses, general practitioners, and specialists on each shift, respectively.  Table 4 shows the cost per hour as contracted for different skills. The additional cost for a nurse, general practitioner, and specialist is 90, 160, and 240 dollars per hour, respectively. The unemployment cost for each one is 50, 70, and 110 dollars per hour, respectively. There are also four holidays a month, and the working duration of full-time, part-time, and hourly contracts is 160, 80, and 40 hours, respectively. Each service provider can work for a maximum of five consecutive days.

### 5.2. Experimental Results

This section describes the experimental results obtained by implementing the proposed approach in the Iranian Health Control Center. The calculations conducted in this case are robust model calculations and two-stage stochastic programming model calculations. The proposed approach is implemented by the GUROBI 9.1(http://www.gurobi.com/) optimization solver on a Macbook pro with an 8-core CPU and an 8 GB RAM.

In the first step, robust model calculations are performed with different values of the conservatism level (Γ).  Figure 3 shows the variation in the conservatism level (Γ) versus the total cost. As can be seen, the total cost increases with an increase in Γ (i.e., when the size of the uncertainty set increases). The results obtained for the total cost and the robustness are presented in Table 5. The robustness value is proportional to the total cost, as determined by the robust optimization and the deterministic method. The total cost remains constant when the conservatism level (Γ) reaches 7.6. In the following, the probability of violating the constraints will be determined by simulation.

Figure 4 illustrates the simulation results for the probability of violating the constraints with 10,000 repetitions. More conservatism leads to increased costs, and the probability of constraint violation is close to zero.

Table 6 presents the probability of constraint violation and a sample of the objective function value. As the protection level rises, the optimal value is marginally affected. For instance, with an increase of the objective function by 6.96%, the probability of constraint violation is just 0.26%.

As shown in Table 6, an increase of Γ raises the total cost to some extent; when the value of Γ reaches 7.6, the total cost remains constant, but there is a rise of 19.38% in it compared to certain conditions. In addition, the robustness value, which represents the status of the objective function, is not high enough to protect against the constraint violation. The computational time for solving the problem is reasonable. Therefore, to solve the model in the next step, a case is considered, in which the cost does not change. With a Γ value of 7.6, the number of service providers is determined for each skill and contract, and the input of the mathematical model becomes known in the next step.

In the second part, the two-stage stochastic programming model is solved based on the results obtained through solving the robust model, which is designed to determine the number of the required service providers. As mentioned in Section 4.2, different methods have been used to cluster scenarios. Based on the initial experiments performed by the SAA method, *N* is 100. Besides, the *N*_k_ (number of clusters) of 20 achieved by clustering methods has yielded better results. Therefore, the model solution is based on these values. In the approach proposed in this study, *N* = 100, *M* = 10 and *N*′ = 20,000 for the original SAA algorithm presented in Section 4.1, and *N*_*k*_=20, *N*_*L*_=1000, *M* = 10 and *N*′ = 20,000 for the I-SAA presented in Section 4.2. These results are reported in Tables 7 and 8. The columns ${\hat{Z}}_{N}^{m}$ and ${\hat{Z}}_{N_{k}}^{m}$ specify the objective function's optimal value considering the *N* and *N*_*k*_ scenarios, respectively. The time column indicates the solution time in seconds. The Gap column shows ${\hat{g}}_{N^{\prime }}\left({\hat{X}}_{N}^{m}\right)-{\bar{Z}}_{N}^{M}$, and the *Var* column shows $S_{{\hat{g}}_{N^{\prime }}\left({\hat{X}}_{N}^{m}\right)}^{2}+S_{{\bar{Z}}_{N}^{M}}^{2}$ for the original SAA. Also, ${\hat{g}}_{N^{\prime }}\left({\hat{X}}_{N_{k}}^{m}\right)-{\bar{Z}}_{N_{k}}^{M}$ and $S_{{\hat{g}}_{N^{\prime }}\left({\hat{X}}_{N_{k}}^{m}\right)}^{2}+S_{{\bar{Z}}_{N_{k}}^{M}}^{2}$ represent the Gap and the Var for the I-SAA, respectively. The original SAA method has the lowest Gap and Var among all the methods. K-means++ has the lowest Gap of the clustering methods, which indicates the most convergence to the optimal solution. Also, the K-means++ method has the lowest mean Var, which denotes the lowest mean-variance of the optimality gap estimate. Next to the k-means++ algorithm, the K-means, PAM, and EM-GMM algorithms have the lowest mean values of Var, respectively.

Figure 5 displays the boxplots of ${\hat{Z}}_{N}^{m}$ for the original SAA algorithm and ${\hat{Z}}_{N_{k}}^{m}$ for the I-SAA. The original SAA algorithm is shown to have the smallest distribution. The K-means algorithm has a small distribution, but it has outliers farther from the mean. The original SAA algorithm has the largest ${\hat{Z}}_{k}^{m}$ of 435995.97 as well as the smallest standard deviation at 878.61. The K-mean++ is the next best algorithm in terms of both ${\hat{Z}}_{k}^{m}$ and standard deviation, with an average of 433530.4 and 1363.28. The EM-GMM and PAM algorithms have the largest standard deviations of 3220.57 and 3663.04, respectively.

In addition, ${\hat{g}}_{N^{\prime }}\left({\hat{X}}_{N}^{m}\right)$ and ${\hat{g}}_{N^{\prime }}\left({\hat{X}}_{N_{k}}^{m}\right)$ are the upper bounds of the optimal solution.  Figure 6 presents the boxplots of ${\hat{g}}_{N^{\prime }}\left({\hat{X}}_{N}^{m}\right)$ for the SAA algorithm and ${\hat{g}}_{N^{\prime }}\left({\hat{X}}_{N_{k}}^{m}\right)$ for the I-SAA with different clustering algorithms. The lowest value of ${\hat{g}}_{N^{\prime }}\left({\hat{X}}_{N_{k}}^{m}\right)$ in the K-means++ method is 437820.84, and the maximum value is 442507.77, which is obtained through the EM-GMM method. There is a 1% change in the upper bound limit.

The highest value of the upper bound is 442507.77, calculated with the EM-GMM, and the lowest value of the lower bound is 422119, obtained through the PAM method. There is a 5% change in the total cost. The results show that K-means++ and the original SAA have yielded the best responses.  Figure 7 illustrates the mean of the upper bound and lower bound of the original SAA and I-SAA with different clustering algorithms. The smallest gap between the mean of upper and lower bounds among the clustering algorithms is 1.5%, which is observed in the K-means++ algorithm. This value for the original SAA algorithm is 0.5%, which has a very small difference from the K-means++ algorithm.

The objective of the SAA algorithm is to reduce computing time. The time taken by the original SAA and I-SAA to solve the SSPSP is also considered to compare the algorithms.  Figure 7 shows the boxplots of the durations for each algorithm to solve the SSPSP for every 10 trials. K-means++ has a better performance than the other algorithms. The K-means and PAM algorithms have the same means, but the K-means++ algorithm has a lower mean and variance. The original SAA algorithm has the slowest run time. The K-means, PAM, and original SAA algorithms have outliers. As Figure 8 suggests, the original SAA algorithm is the slowest, averaging 4.52 seconds. It is also 2.89 seconds slower than the next slowest algorithm, K-means.

The Mann–Whitney test is employed to compare all the solution time means pairwise to determine which ones are significantly different from the rest. The test has been performed on the mean of the solution times, and the results are provided in Table 9. The first and second columns display the algorithm pairs compared. The third column shows the difference between the means. Lastly, the fourth column gives the *p* values for the likelihood of the cases. Considering the significance level of 0.05, there are four cases in which an algorithm in a pair has performed statistically better than the other. All the clustering algorithms are statistically faster than the original SAA algorithm.

Of all the cases, the K-mean++ algorithm shows the best results regarding the solution time and the optimal value. Thus, 431701.5, as the lowest value of the objective function, is selected as the best response. Tables 10–12 show the shift scheduling of nurses, general practitioners, and specialists performed based on the best response obtained. As the tables suggest, morning (MO), afternoon (AF), and night (NI) shifts are specified for each service provider; otherwise, he or she will not be busy.

### 5.3. Managerial Implications

Long-term planning for service providers is one of the most important issues in healthcare organizations. Considering the uncertainties in the demand of patients, especially cancer patients, an appropriate approach to planning is the robust approach, which conservatively determines the number of service providers required. By planning at a strategic level, managers face fewer tactical shortcomings. At the tactical level, where decisions are made to schedule service providers' shifts, managers' power increases to decide on stochastic patients' demands and service providers' working conditions.

In addition to the significant cost reduction resulting from more efficient shift scheduling, the daily use of shift schedules has important managerial implications for the workload of home care, hospital administrators, and service providers. It also frees those individuals to deal with other tasks requiring more direct patient interactions. By setting shift schedules, subjectivity can be excluded from the decisions, and it is possible to use training courses and update the service providers in their free time. Another advantage of this planning is that it provides a robust program against changes in patient demand. Continued use of this plan can be beneficial for patients; necessary predictions have already been made if a shortage of service providers ever occurs. Based on clustered scenarios, managers can also make better decisions in the future. More efficient plans can be made if cooperation between the Iranian Health Control Center and the university continues. Hospitals and other home care centers can use these plans with more required constraints.

## 6. Conclusion

The major contribution of this research is to help healthcare managers specify the minimum number of service providers required. Since service providers' daily and monthly workloads fluctuate, the approach proposed by Bertsimas and Sim [37] has been employed to determine the minimum number of those individuals and solve the proposed SPDP. Based on the most conservative responses obtained in the first step of the research, the number of service providers with different skills and contracts is determined for shift scheduling. Real-world situations in this field often involve different sources of uncertainty, such as patient demand. Among those with this demand for uncertainty, one may refer to cancer patients who experience unpredictable conditions during their illness. Thus, a two-stage stochastic programming model has been presented for shift scheduling, and the SAA and I-SAA methods are used to solve the SSPSP. In the first stage, considering the conservatism level of 7.6, the costs increase by 19.38%, which is shown by the simulation that the probability of constraint violation is zero. In the second stage, this research applies different clustering methods (e.g., K-means, K-means++, PAM, and EM-GMM) to the original SAA method and shows that the K-means++ method obtains a good upper and lower bound of the total cost and achieves a near-optimal solution in the shortest time. Also, the highest value of the upper bound is 442507.77, calculated with the EM-GMM method, and the lowest value of the lower bound is 422119, obtained through the PAM method. It shows just a 5% change in the total costs. Therefore, this research makes the shift program of service providers according to the uncertain patients' demands. A computer-generated provider's schedule is better than a manually generated one to fulfill the task. Apart from the faster scheduling than the manual approach, an important advantage of the proposed approach is that it eliminates subjectivities; no one is involved in providing schedules in the proposed approach, and the level of the available resources is the only factor affecting the final schedule.

Finally, this study presents managerial implications for healthcare authorities who have to solve the problems of dimensioning and scheduling service providers in an uncertain environment.

There are several recommendations for future research in providers' dimensioning and scheduling. The specific skills needed by individual patients can be considered as a basis for assigning relevant service providers. Moreover, the human factors involved in care provision seem interesting topics to study. Other methods can also be tried to solve stochastic programming models. Different robust optimization methods can be applied to providers' dimensioning problems. Disruptive situations can be considered in a model with rescheduling procedures to deal with them. Finally, models may be developed in other areas, such as fire stations and emergency centers, where shift planning is needed.

## Figures and Tables

**Figure 1:** The solution procedures of the two-stage method.

**Figure 2:** Representation of scenario aggregation performed in the I-SSA.

**Figure 3:** The optimal value of the total cost as a function of Γ.

**Figure 4:** Simulation results for the probability of violation.

**Figure 5:** Boxplots of the optimal solution for each algorithm.

**Figure 6:** Boxplots of the upper bound for each algorithm.

**Figure 7:** Mean of the upper bound and the lower bound for each algorithm.

**Figure 8:** Boxplots of the solution time for each algorithm.

**Algorithm 1:** K-means Algorithm.

**Algorithm 2:** K-means++ Algorithm.

**Algorithm 3:** EM-GMM Algorithm.

**Algorithm 4:** PAM Algorithm.

**Table 1:** A brief classification of the models reviewed in the literature.

Author	Year	Service provider dimensioning	Shift scheduling	Objective	Uncertainty	Solution approach
Klinz et al. [17]	2006	—	✓	Minimize the total number of work shifts and the general unhappiness of all nurses	—	Heuristic
Topaloglu and Selim [18]	2010	—	✓	Minimize deviations from nurse preferences and hospital regulations	Fuzzy	Exact
Landa-silva and Le [19]	2008	—	✓	Minimize deviations from nurses' satisfaction and work regulations	—	Meta-heuristic
Ohki [20]	2012	—	✓	Minimize the penalty function to evaluate shift schedules	—	Meta-heuristic
El Adoly et al. [33]	2011	—	✓	Maximize the quality of objectives concerning the importance of constraints	—	Meta-heuristic
Maenhout and Vanhoucke [8]	2013	✓	✓	Minimize the penalty associated with different types of nurses	—	Exact
Santos et al. [22]	2016	—	✓	Minimize the penalty of assignment	—	Heuristic
Ingels and Maenhout [23]	2015	—	✓	Minimize the allocation penalty and change the nurse schedule	—	Exact and simulation
Dohn and Mason [24]	2013	—	✓	Minimize penalties from under-and over-coverage and minimize the total cost of all roster lines	—	Column generation
						Branch and price
Bagheri et al. [25]	2016	—	✓	Minimize the normal and overtime hours of nurses	Stochastic	Sample average
						Approximation
Punnakitikashem et al. [26]	2013	—	✓	Minimize the excess workload on nurses and the cost of staffing	Stochastic	Benders and Lagrangian
Chen et al. [10]	2016	✓	✓	First stage: Minimize the number of nurses. Second stage: Minimize the penalty of the soft constraints of nurses' preferences	—	Exact
Ang et al. [27]	2018	—	✓	Minimize the maximum and average deviations from target nurse-patient ratios	—	Exact
Hamid et al. [28]	2020	—	✓	Minimize the sum of incompatibility among nurses and the total cost of staffing and maximize the satisfaction of nurses with their assigned shifts	—	Meta-heuristic
Pham and Dao [29]	2021	—	✓	Minimize the total cost of assigning nurses to different shifts (morning, evening, night, and day-off)	—	Hybrid metaheuristic
Hassani and Behnamian [30]	2021	—	✓	Minimizing the total cost of allocating shifts to nurses, reserve nurses required, overtime and underemployed costs of a particular type of shift, cost of mismatching the nurse preferences with the roster	Robust scenario-based optimization	Meta-heuristic
Kheiri et al. [31]	2021	—	✓	Minimizing violation of eight soft constraints	—	Hyper-heuristic with statistical Markov model
This study	2022	✓	✓	First stage: minimize the number of service providers. Second stage: minimizes regular work hours, overtime hours, and the cost of idle hours	Stochastic	First stage: exact
						Second stage: improved sample average approximation

**Table 2:** Notations of SPDP.

Sets	
*S*	Set of skills (nurse, general practitioner, and specialist)
*M*	Set of months
*N*	Set of contracts

Parameters	
*d*_*im*_	Demand for skill *i* per month *m*
ca_*jm*_	Contract capacity *j* per month *m*
*a*_*im*_	Number of the service providers available with skill *i* per month *m*
*b*_*jm*_	Number of the service providers available with contract *j* per month *m*
*c*_*ijm*_	Cost of skilled service provider *i* with contract *j*
Γ_*im*_	Conservatism level

Variable	
*x*_*ijm*_	Number of the service providers required for skill *i* with contract *j* per month *m*

**Table 3:** Notations of SSPSP.

Sets	
*S*	Set of skills (xx: nurse, *xy*: general practitioner, and *xz*: specialist)
*W*	Set of weeks
*D*	Set of days
*M*	Set of shifts
*N*	Set of contracts (full time, part-time, and hourly)
*ξ*	Set of scenarios (*ξ*=1,2,…, *B*)
*I*_*xx*_	Set of nurses
*I*_*xy*_	Set of general practitioners
*I*_*xz*_	Set of specialists

Parameters	
*aa*_*ij*_	1, if nurse *i* is under contract *j*
*ab*_*ij*_	1, if general practitioner *i* is under contract *j*
*ac*_*ij*_	1, if specialist *i* is under contract *j*
*h*_*j*_	Number of hours of service by contract *j* per shift
*hh*_*j*_	Number of contract hours *j* per month
*de*_*smd*_	Number of the hours required of skill *s* per shift *m* per day *d*
*ca*_*j*_	Cost of a nurse with contract *j* per hour
*cb*_*j*_	Cost of a general practitioner with contract *j* per hour
*cc*_*j*_	Cost of a specialist with contract *j* per hour
*c*1_*i*_	Additional service cost per hour for skill *i* (*i* *=* *xx*, *xy*, *xz*)
*c*2_*i*_	Penalty cost per hour for working less than the contract for service providers with skill *i* (*i* *=* *xx*, *xy*, *xz*)
*e*1_*s*_	Minimum number of shifts for a full-time service provider with skill *s*
*e*2_*s*_	Maximum number of shifts for a full-time service provider with skill *s*
*n*1	Minimum number of weekends off that a service provider should take in the period
*n*2	Maximum number of night shifts for each service provider
*g*_*i*_	1, if day *i* is weekend

Variables	
*xx*_*imd*_	One if nurse *i* is assigned to shift *m* on day *d*; otherwise, 0
*xy*_imd_	One if general practitioner *i* is assigned to shift *m* on day *d*; otherwise, 0
*xz*_imd_	One if specialist *i* is assigned to shift *m* on day *d*; otherwise, 0
*wx*_*id*_	One if *d* is a working day for nurse *i*; otherwise, 0
*wy*_*id*_	One if *d* is a working day for general practitioner *i*; otherwise, 0
*wz*_*id*_	One if *d* is a working day for specialist *i*; otherwise, 0
*p*_*imd*_^*ξ*^	Number of the additional hours required for skill *i* on shift *m* on day *d*
*q*_*imd*_^*ξ*^	Number of the idle hours for skill *i* on shift *m* on day *d*

**Table 4:** The wage of each skill per hour ($).

	Nurse	General practitioner	Specialist
Full-time	50	60	110
Part-time	60	110	150
Hourly	70	150	200

**Table 5:** Price of robustness.

Γ	Optimal value	Robustness value (%)	Γ	Optimal value	Robustness value (%)
0	4483.2	—	2.7	5059.2	12.8480
0.1	4540.8	1.2848	3.1	5102.4	13.8116
0.3	4564.8	1.8201	3.2	5112	14.0257
0.6	4694.4	4.7109	3.3	5131.2	14.4540
0.9	4718.4	5.2463	3.6	5136	14.5610
1.1	4737.6	5.6745	3.7	5155.2	14.9893
1.2	4795.2	6.9593	3.9	5179.2	15.5246
1.6	4814.4	7.3876	4.6	5208	16.1670
1.7	4838.4	7.9229	4.8	5212.8	16.2741
1.8	4896	9.2077	5.6	5280	17.7730
1.9	4920	9.7430	5.7	5304	18.3084
2	4977.6	11.0278	6.8	5313.6	18.5225
2.1	4982.4	11.1349	7.1	5328	18.8437
2.2	5035.2	12.3126	7.6	5352	19.3790

**Table 6:** Probability of violation.

Γ	Probability of violation	Total cost	Increase (%)	Γ	Probability of violation	Total cost	Increase (%)
0	0.9998	4483.2	—	2.7	0	5059.2	12.85
0.1	0.9927	4540.8	1.28	3.1	0	5102.4	13.81
0.3	0.9906	4564.8	1.82	3.2	0	5112	14.03
0.6	0.4717	4694.4	4.71	3.3	0	5131.2	14.45
0.9	0.4687	4718.4	5.25	3.6	0	5136	14.56
1.1	0.3115	4737.6	5.67	3.7	0	5155.2	14.99
1.2	0.2606	4795.2	6.96	3.9	0	5179.2	15.52
1.6	0	4814.4	7.39	4.6	0	5208	16.17
1.7	0	4838.4	7.92	4.8	0	5212.8	16.27
1.8	0	4896	9.21	5.6	0	5280	17.77
1.9	0	4920	9.74	5.7	0	5304	18.31
2	0	4977.6	11.03	6.8	0	5313.6	18.52
2.1	0	4982.4	11.13	7.1	0	5328	18.84
2.2	0	5035.2	12.31	7.6	0	5352	19.38

**Table 7:** Statistics for each algorithm (${\hat{Z}}_{N}^{m}$ and time).

	SAA		I-SAA							
			K-means		K-means++		EM-GMM		PAM	
*M*	${\hat{Z}}_{N}^{m}$	Time	${\hat{Z}}_{N_{k}}^{m}$	Time	${\hat{Z}}_{N_{k}}^{m}$	Time	${\hat{Z}}_{N_{k}}^{m}$	Time	${\hat{Z}}_{N_{k}}^{m}$	Time
1	436132.5	4.49	429985.5	1.46	434269	1.57	424964.5	1.42	431521.5	1.64
2	437549.7	4.37	430258.5	1.4	432845.5	1.52	430353.5	1.48	425428	1.59
3	436823	4.52	429723.5	1.47	434158.5	1.56	427920.5	1.4	425048.5	1.52
4	436089.7	4.43	428564.5	1.45	434610.0	1.47	426269.5	1.46	428647.5	1.44
5	435876.9	4.56	424405	1.67	434269	1.5	425242	1.45	423996.5	1.75
6	435031.2	4.38	424265.5	2.83	430973.5	1.48	422452.5	1.59	424269.5	1.49
7	435771.1	5.14	427563	1.47	435059	1.42	430550	1.55	427605.5	1.5
8	435976.9	4.4	430788.5	1.48	431701.5	1.48	430101.5	1.54	422119	1.46
9	434353.6	4.43	429696.5	1.55	432895.5	1.51	432737.5	1.49	429652	1.48
10	436355.1	4.5	429849.5	1.53	434522.5	1.53	433758	1.61	431032	1.46

**Table 8:** Statistics for each algorithm (Gap and Var).

	SAA		I-SAA							
			K-means		K-means++		EM-GMM		PAM	
*M*	Gap	Var	Gap	Var	Gap	Var	Gap	Var	Gap	Var
1	2075.25	80444.81	11133.32	568383.3	7851.01	418813.5	11926.14	1344766	14691.07	1040081
2	1961.39	80396.81	10551.23	568258.7	8294.86	418848.3	11051.47	1344891	14744.03	1040044
3	2176.38	80457.34	12884.33	568204.2	6647.68	419070.2	11613.63	1344910	15398.69	1040167
4	1982.29	80502.21	12282.48	568329.2	6510.06	418948.4	14072.82	1344764	12930.52	1040268
5	1903.73	80389.55	11255.07	568203.6	8268.36	418854.7	10050.89	1345136	15007.42	1040214
6	2088.2	80406.9	11495.52	568620.8	6570.52	418978.3	11123.61	1345117	13632.48	1040255
7	2025.16	80484.91	10706.76	568439	4904.69	445945.4	10271.39	1344925	13020.84	1040212
8	1989.42	80422.1	12321.22	568252.2	6783.62	418997	11594.9	1344905	13331.85	1040315
9	2135.13	80453.57	11168.33	568115.2	6474.6	419029.8	11593.65	1344986	14044.61	1040176
10	1887.81	80461.3	10271.09	568299.9	7872.85	419019.8	11875.14	1344871	13728.78	1040055

**Table 9:** Mann–Whitney test on the mean time to solve.

*μ*_1_	*μ*_2_	|diff|	*p* value
Original SAA	K-means++	3.018	0.00018
Original SAA	K-means	2.891	0.00018
Original SAA	PAM	2.891	0.00018
Original SAA	EM-GMM	3.023	0.00018
K-means++	K-means	0.127	0.64903
K-means++	PAM	0.029	0.96977
K-means++	EM-GMM	0.034	0.76193
K-means	PAM	0.098	0.76184
K-means	EM-GMM	0.132	0.87955
PAM	EM-GMM	0.034	0.49515

**Table 10:** Nurses' schedule.

	Days																								
	Nurse number	1	2	3	4	5	6	7	8	9	10	11	12	13	14	15	16	17	18	19	20	21	22	23	24
Full-time	1	AF	NI	AF	MO	MO	—	NI	AF	NI	AF	MO	—	MO	AF	NI	MO	AF	—	NI	AF	NI	AF	AF	—
	2	AF	—	NI	AF	AF	AF	AF	—	AF	NI	AF	NI	MO	—	AF	NI	MO	NI	MO	—	MO	MO	NI	AF
	3	AF	MO	MO	—	AF	NI	AF	NI	AF	—	NI	MO	NI	AF	AF	—	MO	AF	NI	MO	AF	—	NI	AF
	4	NI	MO	MO	NI	—	MO	AF	AF	AF	NI	—	MO	NI	—	MO	AF	NI	MO	MO	—	NI	MO	AF	AF
	5	—	NI	MO	MO	MO	MO	—	NI	MO	AF	MO	MO	—	NI	AF	MO	NI	AF	—	NI	MO	NI	MO	MO
	6	NI	AF	NI	MO	AF	—	NI	MO	MO	MO	AF	—	—	NI	MO	NI	MO	MO	—	AF	MO	AF	MO	NI
	7	—	NI	AF	NI	MO	MO	—	MO	NI	MO	MO	NI	—	MO	MO	NI	AF	AF	—	NI	AF	MO	AF	MO
	8	MO	MO	—	MO	MO	AF	NI	AF	—	MO	MO	NI	AF	NI	—	NI	AF	MO	MO	MO	—	NI	MO	MO
	9	MO	AF	NI	AF	—	MO	MO	NI	AF	AF	—	AF	AF	NI	AF	MO	—	NI	AF	NI	AF	—	NI	MO
	10	NI	AF	MO	NI	—	AF	MO	AF	MO	NI	—	AF	NI	MO	NI	AF	—	MO	AF	AF	AF	NI	—	AF
	11	—	AF	AF	AF	AF	NI	—	NI	MO	AF	AF	AF	—	AF	NI	MO	MO	NI	—	AF	MO	AF	AF	NI
	12	MO	NI	AF	AF	NI	—	MO	MO	NI	MO	NI	—	AF	AF	MO	AF	NI	—	AF	MO	NI	AF	MO	—
Part-time	13	—	AF	MO	—	NI	—	—	—	—	—	—	NI	—	MO	—	—	—	—	—	MO	—	—	—	NI
	14	—	—	—	—	NI	—	—	MO	NI	—	—	—	—	—	—	—	—	NI	—	—	—	—	—	—
	15	—	NI	—	—	—	NI	—	—	—	NI	—	—	—	—	—	—	—	—	—	NI	AF	—	—	—
	16	—	—	—	—	—	—	MO	MO	—	—	—	—	MO	—	—	AF	—	—	—	—	—	—	—	—
	17	—	—	—	—	NI	—	—	—	—	—	NI	—	—	—	NI	—	—	AF	MO	—	—	—	—	—
	18	—	—	NI	—	—	—	AF	—	—	—	—	—	—	—	—	NI	AF	—	NI	—	—	—	—	—
	19	—	—	—	—	NI	AF	AF	—	—	—	—	—	—	—	—	—	—	—	AF	—	—	NI	—	—
	20	AF	MO	—	—	—	—	MO	—	—	—	—	—	—	NI	—	—	AF	—	NI	—	—	—	—	—
	21	—	—	NI	—	—	NI	—	—	—	NI	—	—	NI	—	—	—	—	—	—	NI	—	—	—	—
	22	—	—	—	—	—	NI	—	—	—	—	NI	—	—	—	—	AF	NI	—	MO	—	MO	NI	—	—
	23	—	—	—	—	NI	—	NI	—	—	—	—	—	—	MO	—	AF	—	—	—	—	NI	—	NI	—
	24	—	—	—	—	NI	—	—	—	—	—	—	—	MO	MO	—	—	—	—	—	MO	—	—	—	—
	25	—	—	—	—	—	—	NI	—	—	—	—	—	—	—	MO	—	—	—	—	—	—	—	—	NI
	26	NI	—	—	—	—	NI	—	—	—	—	AF	—	MO	AF	NI	—	—	NI	—	—	—	MO	—	NI
	27	—	—	—	NI	—	—	—	—	—	—	—	AF	—	—	NI	—	—	—	NI	—	NI	—	—	—
	28	—	—	—	—	—	—	—	—	—	—	—	MO	—	—	AF	MO	—	—	—	NI	—	—	—	—
	29	MO	—	—	—	—	AF	—	—	—	—	—	—	AF	—	—	—	MO	AF	AF	AF	—	MO	NI	—
	30	—	—	AF	NI	—	—	—	—	NI	—	NI	—	—	—	—	—	NI	—	NI	—	—	—	—	—

**Table 11:** General practitioners' work schedule.

		Days																							
	General practitioner	1	2	3	4	5	6	7	8	9	10	11	12	13	14	15	16	17	18	19	20	21	22	23	24
	Number																								
**Full-time**	1	MO	AF	NI	AF	——	NI	MO	MO	—	AF	NI	MO	MO	—	NI	AF	AF	AF	MO	—	AF	AF	MO	AF
	2	AF	MO	MO	NI	MO	—	MO	NI	AF	NI	—	NI	AF	MO	MO	NI	—	AF	—	MO	NI	AF	AF	AF
	3	MO	MO	MO	MO	NI	—	NI	AF	MO	MO	AF	—	MO	NI	MO	AF	MO	—	NI	—	NI	MO	NI	MO
	4	AF	AF	NI	MO	AF	—	AF	NI	AF	—	MO	AF	AF	MO	—	MO	AF	MO	AF	NI	—	NI	AF	NI
	5	NI	—	AF	NI	AF	AF	NI	—	MO	AF	AF	AF	—	NI	AF	NI	MO	NI	—	AF	MO	MO	MO	MO
**Part-time**	6	—	NI	—	—	—	NI	—	—	—	—	—	MO	NI	—	—	MO	—	—	NI	—	MO	—	—	—
	7	—	—	—	—	—	MO	AF	—	—	NI	—	—	NI	AF	—	MO	NI	—	—	—	—	—	NI	—
	8	—	NI	—	—	—	MO	—	—	NI	—	NI	—	NI	AF	AF	—	NI	—	—	—	—	—	NI	—
	9	—	—	—	—	—	AF	—	—	—	—	NI	—	—	—	NI	—	NI	—	AF	—	—	—	—	—
	10	—	NI	—	AF	—	MO	—	AF	—	NI	—	—	—	—	—	—	NI	—	MO	—	—	—	—	—
	11	NI	—	AF	—	NI	—	—	AF	—	MO	MO	—	—	—	—	—	—	MO	AF	—	—	—	—	—
	12	—	—	AF	—	MO	AF	—	MO	NI	—	MO	NI	—	—	—	—	—	—	NI	MO	—	NI	—	—
	13	—	NI	—	AF	—	MO	—	—	—	—	—	—	—	—	—	—	—	NI	—	—	—	—	—	NI
	14	—	—	—	—	MO	NI	AF	—	—	MO	—	NI	—	AF	—	—	—	—	—	NI	—	—	—	—
	15	—	—	—	—	NI	—	—	MO	NI	—	—	MO	NI	AF	NI	—	—	NI	—	MO	—	NI	—	—
	16	NI	—	—	—	—	—	—	—	NI	—	—	—	—	—	AF	—	—	MO	MO	AF	AF	—	—	NI

**Table 12:** Specialists' work schedule.

		Days																							
	Specialist number	1	2	3	4	5	6	7	8	9	10	11	12	13	14	15	16	17	18	19	20	21	22	23	24
Full-time	1	AF	NI	MO	—	NI	—	NI	MO	NI	—	MO	—	AF	AF	—	MO	MO	NI	AF	NI	—	MO	AF	AF
	2	MO	NI	MO	AF	—	NI	AF	NI	MO	AF	—	AF	—	—	NI	MO	AF	AF	NI	—	—	NI	MO	MO
	3	NI	MO	AF	NI	—	AF	AF	MO	—	NI	AF	—	—	MO	NI	AF	NI	—	MO	MO	AF	—	NI	MO
	4	—	AF	AF	MO	MO	NI	—	AF	—	MO	—	NI	MO	NI	MO	NI	—	MO	NI	AF	MO	—	NI	AF
	5	—	AF	NI	—	AF	MO	MO	—	AF	—	NI	MO	NI	—	AF	AF	MO	NI	AF	—	NI	AF	AF	NI

## Data Availability

Data are available upon request to the corresponding author.

## References

[1] Zurn P., Dolea C., Barbara S. (2005). World Health Organization Department of Human Resources for Health and International Council of Nurses. *Nurse Retention and Recruitment : Developing a Motivated Workforce*.

[2] Nations U., of Economic D., Affairs S., Division P. (2019). *World Population Ageing 2019: Highlights*.

[3] De Bruecker P., Van den Bergh J., Beliën J., Demeulemeester E. (2015). Workforce planning incorporating skills: state of the art. *European Journal of Operational Research*.

[4] Katholieke S. H., Vives H., de Causmaecker P., Leuven K. U., Lagatie R., Haspeslagh S. (2009). *Negotiation Protocols for Distributed Nurse Rostering*.

[5] Tuna R., Baykal U., Turkmen E., Yildirim A. (2015). Planning for the size of the nursing staff at an outpatient chemotherapy unit. *Clinical Journal of Oncology Nursing*.

[6] Wang W. Y., Gupta D., Potthoff S. (2009). On evaluating the impact of flexibility enhancing strategies on the performance of nurse schedules. *Health Policy*.

[7] De Causmaecker P., Vanden Berghe G. (2011). A categorisation of nurse rostering problems. *Journal of Scheduling*.

[8] Maenhout B., Vanhoucke M. (2013). An integrated nurse staffing and scheduling analysis for longer-term nursing staff allocation problems. *Omega*.

[9] Wright P. D., Mahar S. (2013). Centralized nurse scheduling to simultaneously improve schedule cost and nurse satisfaction. *Omega*.

[10] Chen P. S., Lin Y. J., Peng N. C. (2016). A two-stage method to determine the allocation and scheduling of medical staff in uncertain environments. *Computers & Industrial Engineering*.

[11] Respicio A., Moz M., Pato M. V., Somensi R., Dias Flores C. (2018). A computational application for multi-skill nurse staffing in hospital units. *BMC Medical Informatics and Decision Making*.

[12] Ernst A. T., Jiang H., Krishnamoorthy M., Sier D. (2004). Staff scheduling and rostering: a review of applications, methods and models. *European Journal of Operational Research*.

[13] Cheang B., Li H., Lim A., Rodrigues B. (2003). Nurse rostering problems--a bibliographic survey. *European Journal of Operational Research*.

[14] Viana A. (2011). Operations research in healthcare: a survey. *International Transactions in Operational Research*.

[15] Van den Bergh J., Beliën J., De Bruecker P., Demeulemeester E., De Boeck L. (2013). Personnel scheduling: a literature review. *European Journal of Operational Research*.

[16] Defraeye M., Van Nieuwenhuyse I. (2016). Staffing and scheduling under nonstationary demand for service: a literature review. *Omega*.

[17] Klinz B., Pferschy U., Schauer J. (2006). ILP models for a nurse scheduling problem. *Operations Research Proceeding Operations Research Proceedings 2006*.

[18] Topaloglu S., Selim H. (2010). Nurse scheduling using fuzzy modeling approach. *Fuzzy Sets and Systems*.

[19] Landa-silva D., Le K. N. (2008). A simple evolutionary algorithm with self-adaptation for multi-objective nurse scheduling. *Studies in Computational Intelligence Adaptive and Multilevel Metaheuristics*.

[20] Ohki M. (2012). Effective Operators Using Parallel Processing for Nurse Scheduling by Cooperative Genetic Algorithm. https://www.inderscienceonline.com/doi/abs/10.1504/IJDMMM.2012.045136?journalCode=ijdmmm.

[21] Zhang Z., Hao Z., Huang H. Hybrid swarm-based optimization algorithm of ga & VNS for nurse scheduling problem.

[22] Santos H. G., Toffolo T. A. M., Gomes R. A. M., Ribas S. (2016). Integer programming techniques for the nurse rostering problem. *Annals of Operations Research*.

[23] Ingels J., Maenhout B. (2015). The impact of reserve duties on the robustness of a personnel shift roster: an empirical investigation. *Computers & Operations Research*.

[24] Dohn A., Mason A. (2013). Branch-and-price for staff rostering: an efficient implementation using generic programming and nested column generation. *European Journal of Operational Research*.

[25] Bagheri M., Gholinejad Devin A., Izanloo A. (2016). An application of stochastic programming method for nurse scheduling problem in real word hospital. *Computers & Industrial Engineering*.

[26] Punnakitikashem P., Rosenberber J. M., Buckley-Behan D. F. (2013). A stochastic programming approach for integrated nurse staffing and assignment. *IIE Transactions*.

[27] Ang B. Y., Lam S. W. S., Pasupathy Y., Ong M. E. H. (2018). Nurse workforce scheduling in the emergency department: a sequential decision support system considering multiple objectives. *Journal of Nursing Management*.

[28] Hamid M., Tavakkoli-Moghaddam R., Golpaygani F., Vahedi-Nouri B. (2020). A multi-objective model for a nurse scheduling problem by emphasizing human factors. *Proceedings of the Institution of Mechanical Engineers - Part H: Journal of Engineering in Medicine*.

[29] Pham T. N., Dao S. V. T. (2021). A hybrid metaheuristic algorithm for intelligent nurse scheduling. *Enabling Healthcare 4.0 for Pandemics*.

[30] Hassani M. R., Behnamian J. (2021). A scenario-based robust optimization with a pessimistic approach for nurse rostering problem. *Journal of Combinatorial Optimization*.

[31] Kheiri A., Gretsista A., Keedwell E., Lulli G., Epitropakis M. G., Burke E. K. (2021). A hyper-heuristic approach based upon a hidden Markov model for the multi-stage nurse rostering problem. *Computers & Operations Research*.

[32] Uno A. (2007). BOUNDS for staff size in home help staff SCHEDULING(<Special Issue>the 50th anniversary of the operations research society of Japan). *Journal of the Operations Research Society of Japan*.

[33] El Adoly A. A., Gheith M., Nashat Fors M. (2018). A new formulation and solution for the nurse scheduling problem: a case study in Egypt. *Alexandria Engineering Journal*.

[34] Soyster A. L. (1973). Technical note-convex programming with set-inclusive constraints and applications to inexact linear programming. *Operations Research*.

[35] Ben-Tal A., Nemirovski A. (1998). Robust convex optimization. *Mathematics of Operations Research*.

[36] Sim M. (2004). The price of robustness. *Operations Research*.

[37] Bertsimas D., Sim M. (2001). The Price of Robustness. *Operations Research*.

[38] Birge J., Louveaux F. (2011). *Springer Series in Operations Research and Financial Engineering*.

[39] Kleywegt A. J., Shapiro A., Homem-de-Mello T. (2002). The sample average approximation method for stochastic discrete optimization. *SIAM Journal on Optimization*.

[40] Verweij B., Ahmed S., Kleywegt A., Nemhauser G., Shapiro A. (2001). *The Sample Average Approximation Method Applied to Stochastic Routing Problems*.

[41] Santoso T., Ahmed S., Goetschalckx M., Shapiro A. (2005). A stochastic programming approach for supply chain network design under uncertainty. *European Journal of Operational Research*.

[42] Pagnoncelli B. K., Ahmed S., Shapiro A. (2009). Sample average approximation method for chance constrained programming: theory and applications. *Journal of Optimization Theory and Applications*.

[43] Mak W.-K., Morton D. P., Wood R. K. (1999). Monte Carlo bounding techniques for determining solution quality in stochastic programs. *Operations Research Letters*.

[44] Crainic T. G., Hewitt M., Rei W. (2014). Scenario grouping in a progressive hedging-based meta-heuristic for stochastic network design. *Computers & Operations Research*.

[45] Emelogu A., Chowdhury S., Marufuzzaman M., Bian L., Eksioglu B. (2016). An enhanced sample average approximation method for stochastic optimization. *International Journal of Production Economics*.

[46] Harale M. A., Harale N. D. A survey on clustering in data mining.

[47] Lloyd S. (Mar. 1982). Least squares quantization in PCM. *IEEE Transactions on Information Theory*.

[48] Ostrovsky R., Rabani Y., Schulman L. J., Swamy C. (2012). The effectiveness of Lloyd-type methods for the k-means problem. *Journal of the ACM*.

[49] Dempster A. P., Laird N. M., Rubin D. B. (1977). Maximum Likelihood from Incomplete Data via the EM Algorithm. https://web.mit.edu/6.435/www/Dempster77.pdf.

[50] Kaufmann L. (1987). ClusteringByMedoids_L1Norm_1987. https://www.researchgate.net/profile/Peter-Rousseeuw/publication/243777819_Clustering_by_Means_of_Medoids/links/00b7d531493fad342c000000/Clustering-by-Means-of-Medoids.pdf.

